# Feasibility and Tolerance of Apatinib plus PD-1 Inhibitors for Previously Treated Advanced Gastric Cancer: A Real-World Exploratory Study

**DOI:** 10.1155/2022/4322404

**Published:** 2022-04-29

**Authors:** Li-Hua Li, Wen-Chao Chen, Gang Wu

**Affiliations:** ^1^Editorial Office, Henan Provincial People's Hospital, Zhengzhou University People's Hospital; Henan University People's Hospital, Zhengzhou, Henan 450003, China; ^2^Department of Gastrointestinal Surgery, Henan Provincial People's Hospital; Zhengzhou University People's Hospital; Henan University People's Hospital, Zhengzhou, Henan 450003, China

## Abstract

**Background:**

Apatinib is established to be the standard of care as third-line therapy for patients with previously treated advanced gastric cancer (GC). Programmed cell death protein 1 (PD-1) blockades also exhibited promising efficacy and safety for patients with treatment-refractory advanced GC.

**Objective:**

This study was to explore the feasibility and tolerance of apatinib plus PD-1 inhibitors for patients with previously treated advanced GC.

**Methods:**

This study was performed as a real-world study; patients with advanced GC who were treated with previous systemic chemotherapy were screened retrospectively. Eligible patients were administered with apatinib combined with PD-1 blockade treatment. Efficacy of the patients was assessed with the change of target lesion using radiological evidence according to RECIST 1.1 criteria, and follow-up was carried out regularly. A safety profile was collected and documented during the combination treatment. Univariate analysis based on baseline characteristic subgroup was implemented in univariate analysis to identify the potential factor that might contribute to progression-free survival (PFS).

**Results:**

Between August 2018 and October 2021, a total of 39 patients with advanced GC or gastroesophageal junction adenocarcinoma participated in this study consecutively and all the patients were available for efficacy and safety assessment. The best overall response during apatinib plus PD-1 blockade administration exhibited that PR was observed in 8 patients, SD was noted in 19 patients, and PD was found in 12 patients, which yielded an ORR of 20.5% (95% CI: 9.3%-36.5%), and DCR was 69.2% (95% CI: 52.4%-83.0%). Furthermore, the relatively enough follow-up had resulted in the mature PFS and overall survival (OS) data, suggesting that the median PFS of the 39 patients with advanced GC was 3.9 months (95% CI: 2.74-5.06). Additionally, the median OS of the 39 patients with advanced GC was 7.8 months (95% CI: 4.82-10.78). Furthermore, the most common adverse reactions of the 39 patients who received apatinib plus PD-1 blockades treatment were fatigue (61.5%), nausea and vomiting (56.4%), diarrhea (48.7%), hypertension (46.2%), hand-foot syndrome (38.5%), and rash (28.2%). Furthermore, performance status was independently associated with PFS of apatinib plus PD-1 inhibitor combination administration in baseline characteristic subgroup analysis.

**Conclusion:**

Apatinib plus PD-1 inhibitors exhibited promising effectiveness and acceptable tolerance for previously treated advanced GC preliminarily. And this conclusion should be confirmed in clinical trials in the future.

## 1. Introduction

Gastric cancer (GC), including gastroesophageal junction cancer, was reported to be one of the most common gastrointestinal tumors and the fifth most common malignancy annually all over the world [1]. Specifically, it was reported that there were approximately 1034,000 new cases and 783,000 deaths of GC annually worldwide [2]. And there were almost 479,000 new cases and 374,000 deaths of GC in China currently [3]. Over 95% of GC were diagnosed of adenocarcinomas that were typically classified based on anatomic location and histologic type [4]. And surgery was still the primary therapeutic option for patients with locally advanced GC, and D2 gastrectomy was the standard of care treatment for those who were available for resection [5]. Unfortunately, most patients with GC were diagnosed with metastatic disease initially, and the prognosis remained dismal with a 5-year survival rate of <10% [6]. For those with advanced or metastatic GC, platinum combined with fluoropyrimidine regimens was proved to be the most common first-line treatment, which yielded an objective response rate (ORR) of approximately 40% and median progression- free survival (PFS) and overall survival (OS) of almost 5.5 and 11.5 months, respectively [7]. Amazingly, this year had witnessed that nivolumab plus chemotherapy exhibited a superior OS of over 12 months as the first-line treatment for patients with HER2-negative gastric, gastroesophageal junction, or esophageal adenocarcinoma according to the Check-Mate 649 clinical trial [8]. However, most patients with advanced GC might be refractory to first-line treatment, and the second-line therapeutic options included docetaxel, paclitaxel, irinotecan monotherapy, or the antivascular endothelial growth factor receptor (VEGFR2) antibody ramucirumab alone or in combination with paclitaxel [9]. However, almost all the patients with advanced GC continued to progress in the second-line treatment. And patients were in urgent need of efficacious therapeutic regimens when failed the previous two or more lines of chemotherapy.

A previous study indicated that angiogenesis was associated with a worse prognosis among patients with GC [10]. Therefore, antiangiogenic targeted drugs were developed and demonstrated convincing anticancer activity in the treatment of advanced or metastatic GC [11]. Interestingly, we noticed that ramucirumab (VEGFR2 antibody) monotherapy exhibited convincing effectiveness and acceptable safety profile for patients with metastatic GC according to the RECARD clinical trial [12]. Furthermore, as an oral tyrosine kinase inhibitor (TKI), apatinib selectively bound to and highly inhibited VEGFR2, which had become a novel therapeutic option for patients with advanced or metastatic GC as a third-line treatment in China since 2015 [13]. However, it should be noted that the ORR of apatinib monotherapy was relatively low (ORR = 2.84%), and most treated patients might develop acquired drug resistance ultimately, which highlighted the necessity for new combination strategies.

Interestingly, recent years had witnessed that immunotherapy of PD-1/PD-L1 inhibitors changed the therapeutic landscape of various types of tumors, and unprecedented long-term survivorship was observed for immunotherapy currently [14]. And the previous study indicated that patients with advanced GC were correlated with higher mutation burden and overexpression of immune checkpoint proteins [15]. As a result, recent years had witnessed that PD-1 inhibitors exhibited promising effectiveness and well-tolerated safety profile for patients with GC in both monotherapy and combination therapy consecutively. Nivolumab (PD-1 blockade) monotherapy exhibited a survival benefit as third- or subsequent-line treatment for patients with advanced GC based on the ATTRACTION-2 clinical trial [9]. Additionally, previous work suggested that antiangiogenic TKI plus PD-1/PD-L1 blockades might play a synergistic action in vivo [16]. As a result, PD-L1 blockade plus antiangiogenic targeted drug demonstrated promising efficacy and acceptable safety in the first-line setting among patients with hepatocellular carcinoma [17].

Consequently, this study is aimed at identifying the feasibility and tolerance of apatinib plus PD-1 inhibitors for previously treated advanced GC in the real world.

## 2. Patients and Methods

### 2.1. Study Design

To our knowledge, apatinib and PD-1 inhibitors were approved in China over 3 years, and a considerable number of patients with advanced GC were treated with apatinib plus PD-1 inhibitor administration in clinical practice. As a result, our study was conducted as a real-world study. Patients with advanced GC who received at least one systematic chemotherapy regimen previously in the department of gastrointestinal surgery of Henan Provincial People's Hospital between August 2018 and October 2021 participated in this study retrospectively. And patients with GC met the following criteria were included: (a) histologically confirmed GC or gastroesophageal junction adenocarcinoma with advanced or metastatic stage; (b) aged over 18 years; (c) ECOG PS of 0 or 1 or 2 score; (d) patients were treated with at least one systematic chemotherapy regimens previously; (e) apatinib plus PD-1 inhibitor (any PD-1 blockades that approved in China were permitted) therapy was administered in clinical practice; (f) patients had available measurable target lesion based on the RECIST 1.1 criteria. And the major exclusion criteria were as follows: (a) PD-1, PD-L1, and CTLA-4 blockades or apatinib-based therapy was used previously; (b) consistent with brain metastases that were symptomatic or required treatment; (c) accompanied with autoimmune disease, or patients were diagnosed of immunosuppression and in need of systemic steroid therapy; (d) diagnosed with another cancer or serious diseases; and (e) no available ORR data. Specifically, the study profile is shown in Figure 1. And 39 patients with advanced GC were enrolled ultimately. The protocol of the present study was approved by the ethics committee of Henan Provincial People's Hospital. Written informed consent was provided by each patient enrolled.

### 2.2. Treatment Protocol and Therapeutic Procedures

All the patients included in this study were administered apatinib plus PD-1 inhibitors. Apatinib was used orally with 500 mg or 250 mg once daily continuously, and every 28 days was defined as one treatment cycle. PD-1 inhibitors were any PD-1 inhibitors that were approved in China, which consisted of camrelizumab (200 mg), sintilimab (200 mg), and nivolumab (360 mg). All the three PD-1 inhibitors were intravenously administered according to the previous study [18]. The administration would be terminated when progression or intolerable adverse reactions were observed. When the patients were intolerable to the combination therapy, monotherapy of apatinib or PD-1 blockades was permitted.

Efficacy of the combination therapy was assessed based on RECIST version 1.1 criteria [19]. In detail, radiological scans of the target lesions with CT or MRI were performed before and during the combination therapy individually, which was performed every 6 weeks or might be scheduled ahead of time if there was definite evidence of substantial progression. Additionally, the primary endpoint of the present study was PFS, and secondary endpoints were ORR, disease control rate (DCR), OS and safety profile during the combination administration.

### 2.3. Follow-Up and Adverse Reaction Assessment

When the patients were hospitalized in our department, clinical characteristics and safety profiles were collected from the electronic medical record system. Furthermore, further follow-up was implemented using a mobile phone. Subjects were followed up monthly when progressed the combination treatment to be aware of the death status of the patients. Furthermore, the safety profile of the treatment was assessed using CTCAE 4.03 [20]. The safety profile of the patients who were treated with apatinib plus PD-1 inhibitors was documented, and the maximum toxicity of the patients was recorded to present the toxicity profile.

### 2.4. Statistical Analysis

SPSS version 25.0 (IBM, USA) and Stata version 14.0 were used to analyze and present the data, respectively. Quantitative variables and qualitative variables were presented as median (range) and several patients (percentage), respectively. ORR was defined as the rate of CR and PR among all the patients included. DCR was defined as the rate of CR and PR and SD among all the patients included. Definition of PFS and OS was adopted according to the previous study [13]. The Stata software was used to present the PFS and OS survival curve in univariate analysis. Furthermore, exploratory analysis for potential factors to predict the PFS of the combination regimen was carried out accordingly. Association between PFS and baseline characteristic subgroup was calculated with the log-rank test. *P* < 0.05 was considered suggestive.

## 3. Results

### 3.1. Patients and Tumor Basic Characteristics

The baseline demographic and tumor characteristics of the 39 patients with advanced GC is shown in Table 1. The median age of the 39 patients was 61 years, ranging from 33 years to 80 years. Male and female patients were found in 26 and 13 cases, respectively. Interestingly, gastric cancer was observed in 30 patients, and gastroesophageal junction adenocarcinoma was found in 9 patients. All the patients had adenocarcinoma. Patients with previous treatment of first-line and ≥2 lines were found in 4 and 35 patients, respectively. Most patients were concomitant of >2 metastatic sites (76.9%). Interestingly, apatinib initial dosage of 500 mg and 250 mg was noted in 22 and 17 patients, respectively. Noteworthily, camrelizumab, sintilimab, and nivolumab were used in 26, 8, and 5 patients.

### 3.2. Efficacy of Apatinib plus PD-1 Inhibitor Administration

As we described in the method part, patients whose efficacy assessment data were not available had been excluded from the efficacy analysis. Therefore, efficacy assessments of all the 39 patients with advanced GC were available. The best overall response of the patients indicated that PR was observed in 8 patients (20.5%), SD was noted in 19 patients (48.7%) and PD was found in 12 patients (30.8%), yielding an ORR of 20.5% (95% confidence interval (CI): 9.3%-36.5%) and a DCR of 69.2% (95% CI: 52.4%-83.0%).

Furthermore, the best percentage change in target lesion among the 39 patients who were treated with apatinib plus PD-1 blockade administration is presented in Figure 2. The majority of the target lesions of the 39 patients shrank dramatically. Additionally, the chest CT scan before and after the administration of apatinib plus PD-1 blockades is illustrated in Figure 3, which presented the target lesion in the lymph node of a PR patient. The target lesion in lymph nodes near the stomach fundus responded strikingly after the combined administration of apatinib plus PD-1 blockades, which exhibited that this patient benefited significantly from the treatment of apatinib plus PD-1 inhibitors.

### 3.3. Prognosis of Apatinib plus PD-1 Inhibitor Administration

As we described in the method previously, the data cut-off date of this study was December 15, 2021, and the median follow-up duration from the onset of the combined administration to the date of data cut-off was 7.3 months (follow-up range: 0.2-21.5 months). And there were 3 patients with advanced GC who were still in the treatment at the date of data cut-off. About the PFS data, a total of 33 progression or death events were seen at the date of data cut-off, which yielded the maturity of PFS data with 84.6%. As presented in Figure 4, the median PFS of the 39 patients with advanced GC who received apatinib plus PD-1 blockade administration was 3.9 months (95% CI: 2.74-5.06). Furthermore, the 6-month and 12-month PFS rate was 38.0% (95% CI: 22.9%-52.9%) and 9.6% (95% CI: 2.5%-22.4%), respectively.

Association between PFS and baseline characteristic subgroups was implemented in univariate analysis in order to identify the prognostic significance of baseline characteristic subgroup. And the results are presented in Table 2. Patients benefited from the apatinib plus PD-1 blockade administration uniformly regardless of the baseline characteristic subgroups. Interestingly, it seemed that the ECOG performance status score was correlated with PFS. And the median PFS of patients with ECOG PS of 0-1 score and 2 score was 4.6 months and 2.8 months, respectively (*P* = 0.015). Furthermore, when we analyzed the PFS according to PD-1 blockades separately, camrelizumab, sintilimab, and nivolumab conferred a similar PFS (*P* = 0.427).

Additionally, regarding the OS analysis, a total of 29 death events were observed at the date of data cut-off, which yielded the maturity of OS data with 74.4%. As illustrated in Figure 5, the median OS of the 39 patients with advanced GC who received apatinib plus PD-1 blockade administration was 7.8 months (95% CI: 4.82-10.78). And the 6-month and 12-month OS rate was 61.5% (95% CI: 44.5%-74.7%) and 39.3% (95% CI: 23.6%-54.7%), respectively.

### 3.4. Adverse Reactions of Apatinib plus PD-1 Inhibitor Administration

All the adverse reactions of the 39 patients with advanced GC that occurred during the administration of apatinib plus PD-1 blockades were analyzed and presented. On the whole, treatment-related adverse reactions were observed in 38 patients among the 39 patients included (97.4%). Furthermore, this failed to detect the grade 5 adverse reactions during the combination administration. And the adverse reactions with grades 3-4 were noted in 21 patients among the 39 patients (53.8%). Of the 22 patients who received an initial apatinib dosage of 500 mg, 7 patients required a dosage reduction to 250 mg. About the dose termination of the two drugs, 5 patients (12.8%) experienced a dose termination of apatinib and 3 patients (7.7%) experienced a dose termination of PD-1 inhibitors.

Specifically, as exhibited in Table 3, the common adverse reactions manifested as fatigue (61.5%), nausea and vomiting (56.4%), diarrhea (48.7%), hypertension (46.2%), hand-foot syndrome (HFS, 38.5%), rash (28.2%), AST/ALT elevation (25.6%), proteinuria (20.5%), weight loss (17.9%), reactive cutaneous capillary endothelial proliferation (RCCEP, 15.4%), pneumonia (10.3), and anemia (7.7%). Furthermore, the adverse reactions with grades 3-4 were in the following: fatigue (10.3%), nausea and vomiting (12.8%), diarrhea (7.7), hypertension (12.8%), HFS (10.3%), rash (5.1), AST/ALT elevation (5.1%), proteinuria (5.1%), and RCCEP (2.6%). In general, the toxicity of the 39 patients with advanced GC who were treated with apatinib plus PD-1 blockade administration was acceptable and manageable.

## 4. Discussion

The present study highlighted the feasibility and safety of the administration of apatinib plus PD-1 inhibitors among previously treated advanced GC retrospectively. Collectively, the regimen of apatinib plus PD-1 blockades might be a potentially efficacious and safe therapeutic option for previously treated advanced GC clinically.

Although platinum combined with fluoropyrimidine regimens was proved to be the widely used first-line therapy for patients with advanced or metastatic GC, most patients might progress and develop chemotherapy resistance ultimately. Therefore, the prognosis of advanced or metastatic GC remained disappointing currently [21]. Amazingly, Checkmate 649 and Orient 16 clinical trials had demonstrated that PD-1 (nivolumab and sintilimab) inhibitors combined with chemotherapy might become the standard of care as first-line therapy for patients with advanced GC soon, which were both reported in 2021 [8, 22]. However, neither of the two PD-1 inhibitors had the indication as first-line treatment for patients with advanced GC in China, which meant that not all the patients with advanced GC could choose PD-1 combined with chemotherapy in first-line treatment in China currently. Additionally, the 39 patients included in our study were from August 2018 to October 2021, during this period, and no data regarding PD-1 combined with chemotherapy in the first-line setting was reported and available. Therefore, the regimen of apatinib plus PD-1 inhibitors for patients with previously treated GC was reasonable in our study. A total of 4 patients included in our study were treated with first-line therapy previously. Therefore, most patients in our study had been treated after two lines of the previous administration. As a result, almost all the patients in our study were heavily pretreated chemotherapy-refractory advanced GC. To our knowledge, therapeutic regimens of patients with advanced GC who were chemotherapy-refractory were still limited currently [23]. However, considerable patients with superior physical conditions might need the salvage therapy to improve the OS of patients with GC [24]. Apatinib monotherapy had become the standard therapy for patients with advanced or metastatic GC as the third-line treatment in China since 2015. Additionally, in recent years, we had witnessed that immunotherapy with PD-1 inhibitors also exhibited promising activity and acceptable toxicity for previously treated advanced GC [25]. Therefore, we noticed that nivolumab monotherapy exhibited durable antitumor activity and tolerable toxicity for patients with treatment-refractory GC as the third-line therapy according to the ATTRACTION-2 clinical trial [9]. Unfortunately, it should be noted that an obvious limitation of both apatinib monotherapy and nivolumab monotherapy (PD-1 inhibitors) for patients with advanced GC was the relatively low ORR (<12%), which suggested that the combined administration of apatinib plus PD-1 blockades was of potent importance in this disease.

The combined administration of apatinib plus PD-1 blockades in the present study was reasonable, given that both apatinib and PD-1 blockade (nivolumab) monotherapy had the indications as to the third-line treatment for patients with advanced GC. As a result, the ORR of the 39 patients with advanced GC who received apatinib plus PD-1 blockades at present was 20.5%, DCR was 69.2%, and the median PFS was 3.9 months, which was proved to be an encouraging efficacy and promising PFS numerically. To our knowledge, apatinib inhibited VEGFR-2, PDGFR-*β*, SRC, c-KIT, and RET [26], demonstrating positive clinical outcomes for metastatic GC with ORR of 2.84%, DCR of 42.05%, and median PFS of 2.6 months [13]. Additionally, in real-world settings, previous studies included patients with treatment-refractory advanced GC who received apatinib administration [27]. And the results indicated that the ORR for apatinib single agent among patients with metastatic GC ranged from 5.6% to 8.7%, DCR ranged from 58.3% to 69.6%, and median PFS varied from 2.7 to 4.4 months [28, 29]. Apatinib plus PD-1 blockade combination administration yielded a superior efficacy and PFS than apatinib monotherapy in real-world practice, which suggested that apatinib combined with PD-1 blockades might play a synergistic action to some extent clinically [30]. On the other hand, to our knowledge, six preferred therapeutic regimens were recommended as second-line administration by NCCN guidelines in gastric cancer [31], which yielded the ORR that ranged from 3.8% to 28%, and the median PFS ranged from 2.1 to 4.4 months [32]. Even compared to standard second-line chemotherapy, the efficacy of apatinib plus PD-1 blockades was still comparable and noninferior to the second-line regimens numerically. About the clinical activity of PD-1 blockades, pembrolizumab and nivolumab as monotherapy had been investigated among patients with treatment-refractory advanced GC. Although pembrolizumab demonstrated an ORR of 22% among patients with PD-L1-positive advanced GC according to the Keynote-012 clinical trial, the subsequent trial regarding pembrolizumab among patients with advanced GC failed to show a significant advantage [33]. Additionally, the ATTRACTION-2 study in Asian GC patients who received nivolumab monotherapy demonstrated a dramatical survival benefit, which yielded an ORR of 11.2%, a median PFS of 1.61 months among patients who received 3 mg/kg nivolumab every two weeks [9]. PD-1 inhibitors' single agent for metastatic GC also exhibited a relatively low ORR (<15%). Consequently, clinical outcomes of apatinib plus PD-1 blockades highlighted the synergistic action for cancer therapy, similar to the previous finding in hepatocellular carcinoma patients [17].

Additionally, the potential efficacy predictors of apatinib plus PD-1 blockades in terms of baseline characteristics were also implemented in our study meanwhile. And the results indicated that patients benefited from the apatinib plus PD-1 blockade administration uniformly regardless of the baseline characteristic subgroups. This finding was consistent with previous study initiated by Wang and colleagues [34]. A total of 67 patients with treatment-refractory advanced NSCLC who received anlotinib (another antiangiogenic TKI similar to apatinib) plus PD-1 blockades were included in their retrospective study, and almost all the baseline characteristic subgroup failed to confer a positive association with the PFS of anlotinib plus PD-1 inhibitor administration. However, it should be noted that the performance status score was positively correlated with PFS (*P* = 0.015), the PFS of patients with ECOG PS of 0-1 score was significantly longer than that of patients with PS of 2 scores (median PFS: 4.6 vs. 2.8 months). Therefore, our study suggested that PS of 0 or 1 score might be used as a potential biomarker to predict the PFS of apatinib plus PD-1 blockades. However, this conclusion should be interpreted with caution. To our knowledge, it seemed that patients with ECOG poor scores were associated with a worse prognosis regardless of the therapeutic regimens [18, 35]. Therefore, the conclusion that ECOG performance status might be used as potential biomarker might be elucidated in prospective clinical trials subsequently.

Noteworthily, the follow-up duration of our study was relatively long (median follow-up duration: 7.3 months and range: 0.2-21.5 months), and OS was performed and analyzed in our study accordingly. Amazingly, it seemed that the median OS in our study was better than that of apatinib monotherapy and nivolumab monotherapy (median OS was 6.5 and 5.3 months, respectively) [9, 13]. Interestingly, a previous phase Ia and Ib study initiated by Xu and colleagues recruited 25 patients with chemotherapy-refractory advanced GC or gastroesophageal junction adenocarcinoma who were treated with apatinib combined with camrelizumab (PD-1 inhibitor) therapy, which yielded an ORR of 17.4% and a median PFS and OS of 2.9 and 11.4 months, respectively [11]. Therefore, the efficacy and prognosis of this study were comparable to that of our study. It seemed that the OS of patients with advanced GC had been improved to some extent recently. We speculated the possible interpretation could be attributed to the continued approval of immunotherapy since 2018. Especially, we noticed that nivolumab plus chemotherapy in the first-line treatment demonstrated convincing and improved OS for patients with advanced GC according to Checkmate 649 clinical trial [8]. Additionally, other PD-1 or PD-L1 inhibitors were also available for the patients with advanced GC when they failed the administration of apatinib plus PD-1 blockades, bringing the patients with OS benefits consecutively.

The overall adverse reactions of apatinib plus PD-1 inhibitors were acceptable and manageable, which was in line with the safety profile of the previous study regarding the combination therapy of apatinib plus PD-1 inhibitors among patients with advanced NSCLC [30]. It should be noted that the incidence of grade 3-4 adverse reactions was 53.8%, which was higher than that observed in the study regarding apatinib monotherapy or nivolumab monotherapy for patients with advanced GC (grade 3-4 adverse reactions was approximately 25% and 10%, respectively) [9, 13]. Even though, it seemed that the safety profile of apatinib combined with PD-1 inhibitors was safe for the patients with advanced GC because no grade 5 adverse reaction was detected during the administration of apatinib plus PD-1 blockades. Specifically, the detailed adverse reactions of the combination treatment were fatigue, nausea and vomiting, diarrhea, hand-foot syndrome, rash, AST/ALT elevation, and proteinuria (incidence of >20%), which were in concert with the safety profile of exploratory trial regarding apatinib plus camrelizumab in patients with advanced hepatocellular carcinoma [36]. Other immunotherapy-related adverse reactions such as rash, AST/ALT elevation, RCCEP, and pneumonia were also detected during the combination therapy, which might result from the administration of PD-1 inhibitors [9]. It should be noted that RCCEP was deemed as the specific toxicity of camrelizumab that was administered among 26 patients, which might be slightly lower than that observed for camrelizumab single agent in other cancer (approximately 55%) [37]. The difference suggested that treatment of apatinib might reduce the incidence of RCCEP during camrelizumab administration to some extent. Collectively, the overall adverse reactions of the regimen of apatinib plus PD-1 blockades were acceptable and manageable [38].

Limitations existed in our study inevitably. First of all, the sample size was relatively small as a retrospective study, and only 39 patients were enrolled. The feasibility and tolerability of apatinib plus PD-1 inhibitors were still needed to be validated in more patients. Secondly, PD-1 inhibitors were administered in our study. However, the PD-L1 expression test had not been detected to analyze the association between PD-L1 expression and the efficacy of the combination regimen. Still and all, our study was of clinical guidelines to provide the retrospective medical evidence for apatinib plus PD-1 inhibitors among patients with previously treated advanced GC.

## 5. Conclusion

Our study retrospectively highlighted the feasibility and safety of the combined administration of apatinib combined with PD-1 inhibitors for patients with previously treated advanced GC in the real world, which indicated that apatinib plus PD-1 inhibitor therapy exhibited promising effectiveness acceptable tolerance for patients with previously treated advanced GC preliminarily. And the conclusion should be confirmed in prospective clinical trials subsequently.

## Figures and Tables

**Figure 1:** Study profile regarding apatinib plus PD-1 inhibitors for patients with previously treated advanced gastric cancer.

**Figure 2:** The overall percentage change in target lesion of the 39 patients with advanced gastric cancer who received apatinib plus PD-1 inhibitor administration (gray columns were PR, black columns were SD, and yellow columns were PD).

**Figure 3:** Radiological results of the changes for target lesions in the lymph node of one patient with advanced gastric cancer before and after the administration of apatinib plus camrelizumab.

**Figure 4:** Progression-free survival curve of the 39 patients with advanced gastric cancer who received apatinib plus PD-1 inhibitor administration.

**Figure 5:** Overall survival curve of the 39 patients with advanced gastric cancer who received apatinib plus PD-1 inhibitor administration.

**Table 1:** Patients and tumor basic characteristics.

Characteristic	Total patients (*N* = 39)	Percentage
*Age (years)*		
Median (range)	61 (33-80)	
≥61	21	53.8%
<61	18	46.2%
*Gender*		
Male	26	66.7%
Female	13	33.3%
*ECOG performance status score*		
0-1	25	64.1%
2	14	35.9%
*Primary lesion*		
Gastric	30	76.9%
Gastroesophageal junction	9	23.1%
*Lines of previous treatment*		
1	4	10.3%
≥2	35	89.7%
*Previous targeted drugs therapy*		
Yes	7	17.9%
No	32	82.1%
*History of gastrectomy*		
Yes	17	43.6%
No	22	56.4%
*Number of metastatic sites*		
≤2	9	23.1%
>2	30	76.9%
*HER2 expression status*		
Positive	1	2.6%
Negative	17	43.6%
Not available	21	53.8%
*Initial dosage of apatinib (mg)*		
500	22	56.4%
250	17	43.6%
*PD-1 blockades*		
Camrelizumab	26	66.7%
Sintilimab	8	20.5%
Nivolumab	5	12.8%

Abbreviations: ECOG: Eastern Cooperative Oncology Group; HER2: human epidermal growth factor receptor 2; PD-1: programmed cell death protein 1.

**Table 2:** Univariate analysis of PFS among the 39 patients with advanced GC according to baseline characteristics.

Characteristic	*N*	Median PFS (months)	95% CI	*P*
*Age (years)*				0.439
≥61	21	3.9	2.89-4.91	
<61	18	3.8	2.95-4.65	
*Gender*				0.516
Male	26	3.5	2.67-4.33	
Female	13	4.3	3.03-5.57	
*ECOG performance status score*				0.015
0-1	25	4.6	3.37-5.83	
2	14	2.8	1.89-3.71	
*Primary lesion*				0.539
Gastric	30	4.3	3.24-5.36	
Gastroesophageal junction	9	3.9	2.93-4.87	
*Lines of previous treatment*				0.605
1	4	4.6	3.47-5.73	
≥2	35	3.8	2.77-4.83	
*Previous targeted drugs therapy*				0.637
Yes	7	3.9	2.97-4.83	
No	32	3.7	2.85-4.55	
*History of gastrectomy*				0.447
Yes	17	4.3	3.09-5.51	
No	22	3.8	2.76-4.84	
*Number of metastatic sites*				
≤2	9	4.6	3.46-5.74	0.421
>2	30	3.8	2.98-4.62	
*Initial dosage of apatinib (mg)*				0.417
500	22	4.3	3.13-5.47	
250	17	3.8	2.88-4.72	
*PD-1 blockades*				
Camrelizumab	26	3.9	2.91-4.89	0.427
Sintilimab	8	3.5	2.41-4.59	
Nivolumab	5	4.3	3.27-5.33	

Abbreviations: GC: gastric cancer; ECOG: Eastern Cooperative Oncology Group; PD-1: programmed cell death protein 1.

**Table 3:** Adverse reactions of the 39 patients with advanced GC who received apatinib plus PD-1 blockade administration.

Adverse reactions	Total (*N*, %)	Grades 1-2 (*N*, %)	Grades 3-4 (*N*, %)
Any grade adverse reactions	38 (97.4)		21 (53.8)
Fatigue	24 (61.5)	20 (51.3)	4 (10.3)
Nausea and vomiting	22 (56.4)	17 (43.6)	5 (12.8)
Diarrhea	19 (48.7)	16 (41.0)	3 (7.7)
Hypertension	18 (46.2)	13 (33.3)	5 (12.8)
Hand-foot syndrome	15 (38.5)	11 (28.2)	4 (10.3)
Rash	11 (28.2)	9 (23.1)	2 (5.1)
AST/ALT elevation	10 (25.6)	8 (20.5)	2 (5.1)
Proteinuria	8 (20.5)	6 (15.4)	2 (5.1)
Weight loss	7 (17.9)	7 (17.9)	0 (0.0)
REECP	6 (15.4)	5 (12.8)	1 (2.6)
Pneumonia	4 (10.3)	4 (10.3)	0 (0.0)
Anemia	3 (7.7)	3 (7.7)	0 (0.0)

Abbreviations: GC: gastric cancer; AST: aspartate aminotransferase; ALT: alanine aminotransferase.

## Data Availability

The data generated during this study can be requested from the corresponding authors upon reasonable request.
